# Environmental Factors Involved in the High Incidence of Bladder Cancer in an Industrialized Area in North-Eastern Spain

**DOI:** 10.1155/2022/1051046

**Published:** 2022-07-07

**Authors:** José M. Caballero, Meritxell Pérez-Márquez, José M. Gili, Juan C. Pereira, Alba Gomáriz, Carlos Castillo, Montserrat Martín-Baranera

**Affiliations:** ^1^Department of Urology, Hospital Universitari Mútua Terrassa, Terrassa, Barcelona, Spain; ^2^Department of Paediatrics, Obstetrics & Gynaecology and Preventive Medicine and Public Health, School of Medicine, Autonomous University of Barcelona, Bellaterra, Cerdanyola Del Vallès, Barcelona, Spain; ^3^Department of Urology, Consorci Sanitari de Terrassa, Terrassa, Barcelona, Spain; ^4^Department of Clinical Epidemiology, Consorci Sanitari Integral, Hospitalet de Llobregat, Catalonia, Barcelona, Spain

## Abstract

**Background:**

Bladder cancer (BC) is the most common of those affecting the urinary tract, and a significant proportion of the cases are attributable to tobacco use as well as occupational and environmental factors.

**Objective:**

The aim of this study is to estimate the current incidence of BC in an industrialized area in northeastern Spain and to analyze its time trends over three decades from an ecological perspective.

**Methods:**

Patients diagnosed with histologically confirmed primary BC, during 2018-2019, in an area in northeastern Spain (430,883 inhabitants) were included. Crude and age-standardized incidence rates were estimated per 100,000 person-years based on the number of individuals getting their first diagnosis. An exploratory time trend analysis was carried out to describe the evolution in tobacco use and occupational or environmental risk factors and the incidence of BC in the same area from the 1990s.

**Results:**

295 patients were included (age 72.5 ± 10.3 years; 89.8% men). The crude rate was 62.6 (95% CI: 51.9–73.2) for men and 6.8 (95% CI: 3.4–10.3) for women. The annual rate adjusted to the European Standard Population was 85.3 (95% CI:75.0–95.5) for men and 7.0 (95% CI:4.5–9.5) for women. From 1994 to 2018, the prevalence of smokers decreased in men (42.3% to 30.9%) as well as in the active population working in the industry (44.36% to 22.59%). Nevertheless, the car fleet, especially diesel, has increased considerably. The annual mean concentrations of air (PM_10_, PM_2.5_, O_3_, and NO_2_) and water (nitrates, arsenic, trihalomethanes) pollutants were within the regulatory limit values, but not the maximum levels.

**Conclusions:**

The incidence of BC is one of the highest in men but not in women, despite the decrease in tobacco use and industrial activity (perhaps related to high latency after carcinogen exposure cessation) and despite the control of environmental pollution (the maximum regulatory limit probably needs to be lowered). Finally, a similar exposure to the carcinogen would result in a gender-specific differential incidence.

## 1. Introduction

Bladder cancer (BC) is the most common of those affecting the urinary tract, and the tenth most common cancer in the world, accounting for 3% of all new annual cancer diagnoses. It is four times more frequent in men than in women [1–3]. BC is typical of industrialized areas, being three times more frequent in wealthy areas than in emerging ones, although the highest mortality rates occur in developing countries [4–6]. The highest incidences of BC are observed in Southern Europe, Western Europe, and North America [1–3]. In Spain, in the early 1990s, the crude annual rate of new BC diagnoses was 41.2 per 100,000 men and 6.5 per 100,000 women; when adjusted by age, according to the European Standard Population, the figures were 40.2 in men and 4.8 in women, and according to the Word Standard Population, 27.1 and 2.8, respectively [4, 5]. In the Spanish cancer registry, in 2018, the estimated crude incidence of BC increased to 65.0 for men and 14.7 for women; when adjusted, European and World age-standardized incidence rates were 70.2 in men and 12.5 in women and 27.5 and 5.6, respectively [6].

Previous studies in this industrialized area of the northeast of Spain, Vallès Occidental, demonstrated a high incidence of BC in men: data from 1992 to 1994 showed an annual crude rate for men and women of 44.1 and 6.2 cases per 100,000 person-year, respectively, and an annual incidence adjusted for age to the European Standard Population of 52.2 and 5.4 cases, respectively, per 100,000 person-year [7, 8]. There is no recent study on the incidence of BC in this area, although indirect data suggest that it might be much higher.

Tobacco smoking is the most well-established risk factor for BC, causing 50–65% of male cases and 20–30% of female cases [9]. Occupational exposure is the second most important risk factor for BC. A recent meta-analysis [10] shows that the profile of at-risk occupations has changed over time and may differ for BC incidence. Work-related cases account for 5–25% of all BC cases in men [9–12] due to occupational exposure to carcinogens: aromatic amines in dyestuff manufacture and rubber and other industries are specific agents in the workplace, which have been unequivocally associated with BC. Exposure to polycyclic aromatic hydrocarbons in aluminum process workers and other industries has also been clearly associated with BC. Exposure to industrial oils/cutting fluids, diesel engine exhaust, paints, dyes, chlorinated hydrocarbon solvents, and metals has shown an association with an increased risk in painters, machinists, and other metal workers, workers in the textile industry, printers, hairdressers, dry cleaners, and transport workers [10, 11]. Painters are exposed to solvents and other paint components through inhalation and dermal contact. Thousands of chemical compounds are used in painting products such as pigments, extenders, binders, solvents (toluene, xylene, aliphatic compounds, ketones, alcohols, esters, and glycol ethers), and additives. Hairdressers are exposed to hair dyes and brilliantine (including aromatic amines) and many other compounds such as volatile solvents, propellants, and aerosols, mostly through skin absorption rather than inhalation. However, cohort studies indicated an increased risk for BC among male hairdressers but not among female hairdressers [11].

Moreover, several reports have demonstrated the effects of environmental pollution on BC risk, particularly in water and food supply and arsenic pollution [12–17]. The water contaminants include inorganic arsenic disinfection byproducts that form during water treatment (trihalomethanes) and nitrate [14–16]. Various components of air pollution, including diesel exhaust and polycyclic aromatic hydrocarbons from vehicles and industries, have been shown to contribute to BC [11, 18]. Although it is increasingly evident that there is a genetic susceptibility to BC, its incidence patterns and trends depend on changes in smoking behavior and shifting occupational and environmental regulations.

In the last 30 years, the surgical activity data regarding BC in our area of the northeast of Spain (Vallès Occidental) made us hypothesize that the incidence of BC continued to be among the highest in the world. Since there are no new incidence studies since the 1990s, this study aims to estimate the current incidence of BC cases in the Vallès Occidental healthcare area. Furthermore, as an exploratory objective, time trends over three decades in smoking, occupational, and environmental factors will be described for the same area.

## 2. Materials and Methods

West Vallès Occidental is a highly industrialized and urbanized healthcare area in Catalonia (northeastern Spain) with 430,883 inhabitants (211,784 men and 219,099 women) [19]; public healthcare services rely on two centers, the Hospital Universitari Mútua de Terrassa and the Consorci Sanitari de Terrassa.

From January 1^st^, 2018 to December 31^st^, 2019, all patients admitted in these two hospitals, diagnosed with primary urothelial BC, with histological confirmation, were included in the study. Exclusion criteria were applied for those cases with nonurothelial BC, with a recurrence of a previously diagnosed BC, and for those who were not residents of the study area. Demographic data (age and gender) were recorded. A search was also carried out in the database of the Statistical Institute of Catalonia (IDESCAT) focusing on the habit of smoking, occupation, and environmental pollution in our area in the last 25 years [19].

One of its most important sources of emissions is road traffic, either from the combustion of engines, such as friction and wear of brakes and tires, although they may also be related to other processes in the industrial sector, the agricultural and livestock sector, sector construction, and even within the domestic and service sphere. The Air Quality Index (AQI) is a synthetic indicator prepared from the emission data of the four main primary pollutants for which the current legislation sets the maximum levels: nitrogen oxide (NOx), particles smaller than 10 microns (PM_10_), particles smaller than 2.5 microns (PM_2.5_), and ozone (O_3_). Air pollutants are generally measured in micrograms per cubic meter of air (*μ*g/m^3^). This parameter can take values between -100 (worst quality) and 100 (best quality) [19]. Finally, waters affected by or at risk of contamination include fresh surface water and groundwater that have or may have an excess concentration of nitrates or inorganic arsenic [19–22]. Moreover, although drinking water disinfection is essential for public health, trihalomethanes (THM) are formed at the highest concentrations after chlorination. Total THM concentrations representing the sum of chloroform, bromodichloromethane, dibromochloromethane, and bromoform are the only disinfection byproducts regulated in the European Union (EU) [16, 23]. The maximum regulatory level set by the EU and the World Health Organization (WHO) for each pollutant has changed over the years (Table 1).

This study was approved by the Ethics and Research Committee of the Hospital Universitari Mútua de Terrassa and conformed to the principles of the Declaration of Helsinki.

Statistical analysis was carried out using the SPSS package for Mac, version 21. The annual crude incidence was estimated based on the number of cases registered during the years 2018-2019 at both participating hospitals. For age and gender groups, specific incidence rates were calculated using the 2019 municipal data from IDESCAT as denominators [19]. The direct method was applied to adjust rates for age and gender, using as references the European Standard Population of 2013 [24] and the World Standard Population [25].

## 3. Results

### 3.1. Incidence

The incidence results have previously been published in a preprint [26]. A total number of 295 patients with primary BC were registered during the years 2018 and 2019 : 155 cases (52.5%) at the Hospital Universitari Mútua de Terrassa and 140 cases (47.4%) at the Consorci Sanitari de Terrassa. The annual global incidence per 100,000 person-year was 34.2 cases (95%CI: 30.3–38.1); 62.6 cases (95%CI: 51.9–73.2) in men and 6.8 cases (95%CI: 3.4–10.3) in women. The annual rate adjusted to the European Standard Population was 41.2 (95% CI: 36.5, 45.9) and to the World Standard Population was 15.9 (95% CI: 13.0–17.8). When analyzed by gender, the annual incidence adjusted to the European Standard Population was 85.3 (95% CI: 75.0–95.5) in men and 7.0 cases (95% CI: 4.5–9.5) in women, and 31.7 (95% CI: 27.9–35.5) and 2.9 (95% CI: 1.8–3.9), respectively, when adjusted to the World Standard Population.

The number of BC cases in 2018 and their crude and adjusted rates in our area under study (West Vallès Occidental) compared to several European countries are presented in Table 2 [6, 27]. The crude annual incidence in our area was very high in men (62.6), this indicator being similar to the one in Spain (65.0), but becoming higher when adjusted to the European Standard Population (85.3 vs 70.2) or the World Standard Population (31.7 vs 27.5) [6, 27].

The incidence rate in men adjusted to the World Standard Population in our area under study was much higher than that in other areas of the world and ranked third, after Greece and Lebanon when compared to the countries with the highest BC incidence rates in men [28]. On the other hand, in women, in 2018, the incidence rate adjusted to the World Standard Population was the lowest when compared to the countries with the highest incidence in men [28]. In our area of the northeast of Spain, the incidence of BC in men, adjusted to the European Standard Population, ranks second after Greece among the European countries, with a much lower incidence in women (Table 2) [6, 27].

### 3.2. Demographic Data

The mean age was 72.5 years (SD = 10.4; range 30–91 years), and 89.8% were male, with no statistically significant differences in the mean age between genders. According to the age distribution, 77.3% of the patients were over 65 years (78.1% of men and 70.0% of women). BC was rare at younger ages, since only 6 patients (2.0%) were under 50 years. The highest crude annual incidence rate was observed in the 80–84 years age group for the entire sample; in the 75–79 age group for men, and the 85 to 89 age group for women (Table 3) [19].

### 3.3. Time Trends in Risk Factors

#### 3.3.1. Smoking

In Catalonia, in 1994, the prevalence of smokers in the population over 15 years of age was 42.3% in men and 20.7% in women. In 2018, the prevalence in men decreased to 30.9, although it was still high in the 35–44 age group (40.3%). However, in 2018, the prevalence of smoking remained in women (20.5%), the highest being between 25 and 34 years (31.6%) [19]. Previous studies showed that 84.9% of BC cases diagnosed during 1993–1995 in the Vallès Occidental had ever smoked [29]. In the current study, 179 of 295 BC cases diagnosed during 2018–2019 were smokers, which represents a decrease to 60.7%.

#### 3.3.2. Occupational Exposure

In 1994, 44.36% of the total active population in the Vallès Occidental worked in industries and 48.49% in services. Over the years, the population employed in the industry decreased to 22.59% at the expense of an increase in the population working in services to 72.24% (Figure 1) [19]. In the 1990s, the two industrial activities with more workers, with a considerable difference over the rest, were those of metallurgy and metal products and that of textiles, clothing, leather, and footwear, but in the following years, both suffered a sharp drop in employment, more accused in the case of the textile that in the one of the metallurgy. Indeed, in the period 2000–2018, the textile industry lost 62.6% of its workforce, while in metallurgy, the decrease was 34.3% [19, 30]. However, in 2017, there were 170 industrial estate zones in the Vallès Occidental, of which 21.5% were created in the period 1991–2000 and 16.9% in the period 2000–2017. This area of northeast Spain, Vallès Occidental, has therefore the largest total area of an industrial zone in Catalonia (4,700 hectares) [19, 30]. Regarding the typology, it should be noted that an important part belongs to the chemical industry and waste management (both represent 29%), followed by the metallurgical industry (18%) and the agri-food industry (10%). Other minority types in the region would be the mineral industry (8%), the one related to the consumption of organic solvents (5%), and the paper, cardboard, and wood derivatives industry (1%) [30].

#### 3.3.3. Environmental Air Carcinogens

Due to the industrial activity and the large volume of road traffic that circulates every day in and around the municipalities of our study area, this region has levels of NOx and particles (PM_10_ and PM_2.5_) above those recommended by WHO to preserve the health conditions of the population [19].

All types of vehicles have increased in number between 1997 and 2019 [19]. In addition, when analyzing the increase in the number of vehicles between 2010 and 2019 in the Vallès Occidental according to fuel, it has been higher in diesel vehicles (from 268,805 to 298,492) than in gasoline vehicles (from 308,115 to 318,503) [19].

When analyzing the average of the maximum, minimum, and mean values of the AQI of the stations in the Vallès Occidental, from 2001 to 2019, air pollution showed a worsening, especially in the minimum values (from 4.3 in 2001 to −71 in 2019) [19]. When comparing the annual mean urban levels of the four pollutants that determine AQI of the West Vallès occidental (Terrassa and Rubi stations) with the European urban averages, we observed that in the study area, the levels of O_3_ and NO_2_ were higher while those of PM_2.5_ were similar and those of PM1_0_, lower (Figure 2) [31].

In the period 2010–2020, the annual limit value of NO_2_ (40 *μ*g/m^3^ by EU and WHO) was exceeded in several stations in the West Vallès Occidental, especially in the capital of the area (Terrassa). For suspended particles (PM_10_), the normative annual limit value (40 *μ*g/m^3^) has never exceeded since 2010, whereas the limit set by the WHO (20 *μ*g/m^3^) has been overstepped at all control stations in the study area. In recent years, although there has been no exceedance of the PM_2.5_ limit value according to current regulations (25 *μ*g/m^3^ by EU), the value set by the WHO has been exceeded every single year (10 *μ*g/m^3^) at all stations in the study area [19]. Finally, the annual average O_3_ concentration in recent years has been between 32 and 56 *μ*g/m^3^ at Vallès Occidental stations. In relation to the 8-hour maximums, the limit values set by the regulations have been exceeded each year currently (120 *μ*g/m^3^) at most stations, and by 2018, at all stations. On the other hand, in relation to health, the value set by the WHO (100 *μ*g/m^3^) has been exceeded every year at almost all stations [19].

#### 3.3.4. Environmental Carcinogens in Water

From the analysis of nitrate concentration of groundwater in the Vallès Occidental (Figure 3), the authors of [21, 22] set the quality standard at 50 mg/L, percentile 50 values range from 35 to 64 mg/L and the maximum values detected in each of the annual series were always above 100 mg/L. In general, between 48.4 and 70% of the samples analyzed were above the quality standard (50 mg/L), except in 2007 (33.3%) and 2008 (17.9%). The graphs show the evolution of the concentrations with a possible upward trend; in any case, in general terms, no improvement is observed in groundwater quality [21, 22]. For the above, the EU has declared the Vallès Occidental as a vulnerable zone (all those zones draining into waters that are or could be affected by high nitrate levels) [22].

Inorganic arsenic is naturally present at high levels in the groundwater. Drinking water crops irrigated with contaminated water and food prepared with contaminated water are the sources of exposure. The presence of arsenic in groundwater comprises a worldwide problem in the EU, where many countries are affected by elevated arsenic concentrations (i.e., Greece, Hungary, Romania, Croatia, Serbia, Turkey, and Spain) [32]. Data on the arsenic valuation of each of the three water bodies of West Vallès Occidental (Prelitoral Castellar de Vallès, Al.luvials del Vallès, and Ventall al.luvial de Terrassa) were obtained from the information collected in several monitoring points located in each of the water bodies [20]. In the period 2008–2018 (no data for 2012), the mean concentration of arsenic in groundwater in the West Vallès Occidental (annual average samples = 42.5) decreased, but the mean concentration was 2.66 *μ*g/L, which is higher than the mean concentration reported by Spain in the same period (0.77 *μ*g/L) (Figure 4) [20, 33]. The percentage of water bodies in a good status for arsenic values was 96.43% (92.18–100%) for West Vallès Occidental vs 99.19% (99.06–99.30%) for Spain [20, 33]. Of a total of 435 samples from the 2008–2018 period in the West Vallès Occidental, there were 23 samples (5.3%) with arsenic levels in the groundwater higher than 10 *μ*g/L (mean = 23.87 *μ*g/L; range 15.00–41.00 *μ*g/L) [20].

Furthermore, inorganic arsenic is found mainly in plants because they can absorb arsenic from contaminated soil or water. In Catalonia, the analysis of inorganic arsenic concentrations in 70 types of food between the years 2000 and 2017 shows a very significant reduction, although it is difficult to make comparisons because in studies before 2012, it was calculated by means of an estimate; however, from 2012, it is analyzed particularly: the mean intake of inorganic arsenic in µg/day in the years 2000, 2005, 2008, 2012, and 2017 was 42.42, 16.90, 27.38, 3.48, and 2.58, respectively. The foods that had the highest concentrations of inorganic arsenic were bread and cereals and their derivatives, but they did not exceed the legal limits. In recent years, the values calculated for various groups of the Catalan population are found below the established toxicological safety level (0.3–8 *μ*g/kg/day); however, the resulting margins of exposure are small and cannot be ruled out a completely certain health risk [34].

THM is a widespread disinfection byproduct in drinking water, and long-term exposure has been consistently associated with increased BC risk. The THM levels in drinking water of 26 countries of the EU in the period 2015–2018 described that the highest mean THM values were observed in Cyprus (66.2 *μ*g/L), Malta (49.4 *μ*g/L), Ireland (47.3 *μ*g/L), Spain (28.8 *μ*g/L), and Greece (26.3 *μ*g/L). Maximum reported concentrations exceeded the EU regulatory limit for 9 of the 22 countries with available data, including Spain with a maximum value of 439.0 *μ*g/L. The estimated annual BC cases attributable to THM exposure ranged from zero in Denmark to 1,482 in Spain [16]. The annual mean THM level in the waters of West Vallès Occidental in the last three years (2019–2021) was 33.39 *μ*g/L, higher than the levels of Spain, but with a maximum value of 75.0 *μ*g/L [23].

## 4. Discussion

The incidence of BC in the studied area of the northeast of Spain was very high in men, as reported in previous studies [7, 8]. When considering the crude annual rate, such a figure was similar to the one in Spain for the same period but became higher when adjusting to the European or World Standard Populations [6, 27, 28]. When compared with all European countries, in 2018, the incidence of BC in men, adjusted to the European Standard Population, ranked second after Greece [6, 27] and third after Greece and Lebanon when adjusted to the world population [28]. Alternatively, the incidence in women was much lower, ranking the lowest of all European countries whether considering the crude or the adjusted rate (European Standard Population) and was one of the lowest when considering the incidence adjusted to the World Standard Population [4, 5, 7].

According to the previously published incidence of BC in Vallès Occidental during the period 1992–1994, both the crude and age-adjusted annual incidence has risen in both sexes, although the increase in men is notably higher [7, 8]. The high incidence of BC in men, about 25 years later, could be related to a high prevalence in this area of well-known risk factors for BC, such as smoking, residence in industrialized areas, and occupational exposure to certain carcinogenic products [8, 29].

Advanced age and male sex contribute to the development of BC but are clearly nonmodifiable risk factors. Tobacco consumption is a well-established risk factor for BC. Although data on tobacco consumption are not available in Vallès Occidental, the figures obtained for Catalonia can be extrapolated. The fact that between 1994 and 2018, smoking decreased in men and remained unchanged in women points to other risk factors involved in BC. Former smokers have a lower risk of BC compared with current smokers, but findings on the dose-response relationship between years after quitting smoking and the risk of bladder cancer are inconsistent. Recently, the European Association of Urology (EAU) guidelines estimated a 40% reduction in the risk of developing BC within 1–4 years of quitting smoking, increasing to a 60% reduction after 25 years of smoking cessation [9]. However, the relative risk was still 50% increased after 20 years of cessation, although the risk decreased with longer cessation of cigarette smoking, equally in men and women [35].

Occupational exposure is the second most important risk factor for BC and it is likely to occur in occupations in which dyes, rubbers and textiles, paints, leathers, and chemicals are used. From 1994 to 2019, the active population working in the industry in Vallès Occidental has decreased at the expense of the service sector. Although the population working in the industrial sector has decreased, the Vallès Occidental continues to be the most industrialized area of Catalonia. Historically, the high incidence of BC in the Vallès Occidental area was related to the existence of an important textile industry since the mid-19th century. The decline of the textile industry began in the 1970s, becoming marginal at the end of the eighties. In the 1992–1994 studies, when a high incidence was observed, only found some moderate occupational risk in relation to previous and prolonged exposures in the textile industry [8, 29] as a significant percentage of the population had previously worked in this sector without the current security conditions. The EAU guidelines [9] describe that the risk of BC due to occupational exposure to carcinogenic aromatic amines is significantly greater after ten years or more of exposure; the mean latency period usually exceeds 30 years. Population-based studies established the occupational attribution for BC in men to be 7.1%, while no such attribution was discernible for women. Our study shows that more than three decades after the receding of the textile industry, the incidence of BC in men has not decreased, and it is higher than before, especially in patients over 70 years of age. Therefore, although smoking and occupational exposure are the most important risk factors for BC, the decrease in tobacco use in men and the decline of the industrial sector (especially, the textile industry), is not associated with a decrease in the incidence of BC. This may be due in part to the high risk of BC even 30 years after cessation of smoking or occupational carcinogen exposure, as most BC are diagnosed at an advanced age. Perhaps, it would take more years for smoking and occupational exposure cessation to influence the overall incidence of BC.

Furthermore, there are other factors that can also contribute to the high incidence of BC in Vallès Occidental, which are probably related to groundwater contamination with arsenic and THMs, and less likely with nitrates. First, although the annual arsenic groundwater concentration in this area was lower than 10 *μ*g/L, from 2008 to 2018, 5.3% of the analyzed samples showed higher levels. A meta-analysis suggests that exposure to 10 *μ*g/L of arsenic in drinking water may double the risk of bladder cancer, or at the very least, increase it by about 40% [14]. Second, the annual mean THM levels in the waters of West Vallès Occidental in the last three years were 33.39 *μ*g/L, with a maximum value of 75.0 *μ*g/L. Although the maximum regulatory limit established is 100 *μ*g/L, men exposed to annual mean THM levels >25 *μ*g/L had a 35% increased BC risk, and those exposed to >50 *μ*g/L had a 51% increased risk compared to levels <5 *μ*g/L [36]. Finally, the presence of nitrogen compounds (especially nitrates) is the most important problem of diffuse pollution in the groundwater of Catalonia: 50% of groundwater bodies have been declared in poor chemical condition, of which 83% have been diagnosed with excess nitrates. Thus, excess nitrates cause a poor condition in 41% of water bodies underground in Catalonia [21, 22]. Epidemiologic evidence for an association between drinking water nitrate and BC is mixed, but a recent study suggests that nitrate concentrations in drinking water below the current regulatory limit are associated with BC, and these associations may be stronger among those with higher red or processed red meat consumption [15].

In relation to environmental air carcinogens, the AQI has worsened in relation to the minimum values when compared with the European urban averages, apparently at the expense of O_3_ and NO_2_. The car fleet has increased considerably, mainly at the expense of diesel vehicles, and the pollutants NO_2_, PM_10_, PM_2.5_, and O_3_ may affect the health of the exposed population of the region. The latter is a secondary pollutant related to nitrogen oxides, which can become problematic at high concentrations and in atmospheric conditions of high solar radiation and low dispersion [19]. Although a recent meta-analysis described that the quality of evidence on the association between air pollutants and bladder cancer was low or very low, the authors of the publication raised their concern about the validity of the conclusions because of the heterogeneity of the study designs. The currently available evidence on the association of BC and air pollution comes mostly from occupational environments, for example, in motor vehicle drivers, who are occupationally exposed to a considerable amount of traffic-related air pollution. However, even if the intensity of air pollution exposure in the general population is considerably lower than for drivers, it is reasonable to suppose that a lifetime exposure to air pollution could be associated with an increased risk of urinary tract cancer in the general population [17]. A growing body of evidence supporting a wide range of acute and chronic effects on health, including BC, has led WHO to lower the advisory limits for the concentration of air pollutants in 2021.

The mean age of BC diagnosis was similar to the one reported in the other series [7, 37, 38], without differences between both genders. As in the previous study [7], the incidence of this cancer in Vallès Occidental is ten times higher in men than in women, while in the World Population, it is only four times higher. The discrepancy in incidence between genders in different countries has been attributed to differences in the prevalence of tobacco use. Thus, countries like Lebanon, where smoking is culturally prevalent among women, have the highest incidence of BC [1–3]. Other factors that may reduce women's predisposition to BC would be those related to hormonal and genetic factors and lower occupational exposure to carcinogenic products in agriculture, textile, chemical, or construction industries [10–12, 39, 40]. Certain dietary habits such as the consumption of coffee and alcohol, low consumption of fruits and vegetables, and diets rich in red meat and animal proteins are factors possibly implicated in the higher incidence in men than in women [9, 10, 12, 29, 35]. However, other authors consider that the gender difference in BC incidence is independent of the differences in exposure risk, including smoking status [41]. Potential molecular mechanisms include a different metabolism of carcinogens by hepatic enzymes between men and women, resulting in differential exposure of the urothelium to carcinogens. The glutathione-S-transferase M1 and uridine 50-diphosphoglucuronosyltransferase are two of the hepatic enzymes involved in the metabolism of foreign substances; they modulate the exposure of bladder urothelium to carcinogens and therefore influence BC risk. Differences observed between men and women in the expression of these enzymes may result in differences in metabolic processing and consequently, differences in the exposure of the urothelium to carcinogens. According to this hypothesis, similar exposure to a carcinogen would result in a differential gender-specific incidence of BC. In addition, the activity of the sex steroid hormone pathway may play a role in BC development, partly explaining the gender differences: a higher androgen-mediated susceptibility of BC cells to carcinogens and the biologic effects of androgens and estrogens in BC in vitro and in vivo [41].

## 5. Conclusions

The incidence of BC in this industrialized area of northeastern Spain remains one of the highest in men and one of the lowest in women, both in the EU and in the world, despite the decrease in tobacco use and industrial activity. The annual mean concentrations of air and water pollutants were within the regulatory limit values. However, the maximum levels detected used to be above these limits. A longer latency after cessation of exposure to the carcinogen (tobacco and industry) and a better control of air and water pollution may be needed, which would mean lowering the maximum permissible pollutant limits. Finally, similar exposure to the carcinogen would result in a gender-specific differential incidence. Therefore, a case-control study would be valuable to identify the risk factors specifically related to BC in this area.

## Figures and Tables

**Figure 1:** Percentage of the population affiliated with the National System of Health by occupational sectors (farming, industry, construction, and services) from 1994 to 2019 in Vallès Occidental [19].

**Figure 2:** Air pollutants' annual mean concentration (O_3_, NO_2_, PM_2.5_, PM_10_) in West Vallès Occidental and European Union (EU) from 2001 to 2019 (PM_2.5_ since 2007) [19, 31].

**Figure 3:** Data per year of the analysis of nitrates (mg/l) in the water samples of our sanitary area from 2002 to 2019 [21, 22].

**Figure 4:** The annual mean of arsenic water concentration (*μ*g/L) in the groundwater samples of Spain and West Vallès Occidental from 2008 to 2018 [20, 33].

**Table 1:** Evolution of the maximum regulatory level set by the European Union (EU) and the World Health Organization (WHO) for each pollutant.

Pollutant		Regulatory level EU		Regulatory level WHO	
Air concentration		(EU, 1999)^*∗*^^1^	(EU, 2008)^*∗*^^2^	(WHO, 2006)^#1^	(WHO, 2021)^#2^
PM_2.5_ *μ*g/m^3^	Annual 24-hour^a^	25	20	10	5
				25	15
PM_10_ *μ*g/m^3^	Annual 24-hour^a^	40	40	20	15
		50^C^		50	45
NO_2_ *μ*g/m^3^	Annual 1-hour 24-hour^a^	40	40	40	10
		200		200	
					25
O_3_ *μ*g/m^3^	Annual 8-hour^b^				60
		120^*∗*^^3^	120	100	100

Water concentration		(EU, 1998)^*∗*^^4^	(EU, 2020)^*∗*^^5^	(WHO, 2008)^#3^	(WHO, 2017)^#4^

Arsenic *μ*g/L	Annual	10	10	10	10
Nitrate mg/L	Annual	50	50	50	50
Trihalomethanes total *μ*g/L	Annual	100	100	100	100

EU = European Union; WHO = World Health Organization.^a^99^th^ percentile (i.e., 3-4 exceedance days per year).^b^Average of daily maximum 8-hour mean concentration. ^c^Not to be exceeded more than 35 times a calendar year × ^∗1^ Council Directive 1999/30/EC of 22 April, 1999, relating to limit values for sulfur dioxide, nitrogen dioxide, and oxides of nitrogen, particulate matter, and lead in ambient air. ^*∗*^^2^Directive 2008/50/EC of the European Parliament and of the Council of 21 May 2008 on ambient air quality and cleaner air for Europe. (OJ *L* 152, 11.6.2008, pp. 1–44) ^*∗*^^3^Directive 2002/3/EC of the European Parliament and of the Council of 12 February 2002 relating to ozone in ambient air. ^*∗*^^4^Council Directive 98/83/EC of 3 November 1998 on the quality of water intended for human consumption ^*∗*^^5^Directive (EU) 2020/2184 of the European Parliament and of the Council of 16 December 2020 on the quality of water intended for human consumption (recast). ^#1^WHO Air quality guidelines for particulate matter, ozone, nitrogen dioxide, and sulfur dioxide. Global update 2005. Summary of risk assessment. Geneva: World Health Organization; 2006. ^#2^WHO global air quality guidelines. Particulate matter (PM2.5 and PM10), ozone, nitrogen dioxide, sulfur dioxide, and carbon monoxide. Geneva: World Health Organization; 2021. ^#3^Guidelines for drinking water quality (electronic resource): incorporating the 1st and 2nd addenda, Vol.1, recommendations. 3^rd^ ed. Geneva: World Health Organization; 2008. ^#4^Guidelines for drinking water quality: the fourth edition incorporating the first addendum. Geneva: World Health Organization; 2017.

**Table 2:** Number of cases and estimated incidence of bladder cancer, crude and age adjusted to the European Standard Population and the World Standard Population, in European countries in 2018, compared to the study area.

Countries	Men				Women			
	N	CR	AIe	AIm	N	CR	AIe	AIm
Germany	27,812	68.6	66.6	26.4	7,926	19.0	15.1	6.3
Austria	984	22.9	25.1	9.9	370	8.3	7.3	3.0
Belgium	3,503	61.7	70.2	27.7	955	16.4	15.1	6.4
Bulgaria	1,448	42.3	44.5	20.8	438	12.1	10.3	4.9
Cyprus	121	20.3	30.2	12.4	43	7.2	9.0	3.9
Croatia	994	49.5	55.5	23.4	346	16.0	13.7	6.1
Denmark	1,954	68.3	74.4	29.3	570	19.7	18.6	7.7
Slovakia	842	31.8	45.7	18.5	324	11.6	12.0	5.2
Slovenia	388	37.5	42.1	16.9	137	13.1	11.3	5.0
Spain	14,793	65.0	70.2	27.5	3,475	14.7	12.5	5.6
Estonia	201	32.8	42.4	16.7	78	11.2	9.1	3.9
Finland	947	34.6	36.9	14.0	245	8.7	7.3	2.8
France	13,408	41.8	45.6	17.2	2,874	8.7	7.3	2.7
Greece	5,106	93.1	95.1	40.4	694	12.3	10.4	4.5
Hungary	2,334	50.6	60.9	26.9	1,057	20.8	18.7	9.1
Ireland	680	28.5	41.8	15.8	260	10.7	13.5	5.5
Iceland	69	40.7	53.6	22.1	17	10.1	11.9	5.3
Italy	20,695	71.6	66.2	27.4	5,213	17.2	13.3	6.0
Latvia	361	40.7	51.3	21.1	167	16.0	13.1	5.9
Lithuania	425	32.1	41.3	16.3	157	10.1	8.2	3.4
Luxembourg	89	30.0	44.6	15.3	21	7.2	8.3	2.7
Malta	106	48.8	54.3	21.6	27	12.6	11.6	4.6
Norway	1,182	43.7	55.1	20.9	371	14.0	14.8	5.9
Netherlands	5,087	59.8	66.1	25.8	1,628	19.0	18.0	7.9
Poland	8,197	44.5	56.8	23.7	2,686	13.6	12.9	5.8
Portugal	1,765	36.2	36.0	14.6	575	10.6	8.3	3.1
United Kingdom	8,826	26.9	30.6	10.8	3,392	10.1	9.6	3.6
Czech Republic	2,169	41.5	49.5	19.8	774	14.3	13.1	5.2
Rumania	3,051	32.2	38.5	16.9	873	8.6	8.0	3.3
Sweden	2,177	43.6	46.8	17.8	682	13.7	12.7	5.1
Study area West Vallès Occidental	133	62.6	85.3	31.7	15	6.8	7.0	2.9
EU28	128,463	51.4	55.4	22.0	35,987	13.8	12.1	5.1
EU28 + EFTA	131,751	51.3	55.4	22.0	36,951	13.8	12.1	5.1

N: number of cases. CR: crude incidence rate. AIm: incidence adjusted to the Word Standard Population. AIe: incidence adjusted to the European Standard Population, 2013 (EU28 + EFTA). All incidence estimations are expressed per 100,000 people year. Sources [6, 27]: ECIS, 2020; REDECAN, 2019.

**Table 3:** The crude incidence rate of BC stratified by age and gender according to the population of West Vallès Occidental in 2018-2019 [19].

	Men			Women		
	Population (inhabitants)	N	CR	Population (inhabitants)	N	CR
0–4 yrs	11,424	0		10,662	0	
5–9 yrs	13,568	0		12,665	0	
10–14 yrs	14,195	0		13,524	0	
15–19 yrs	12,660	0		11,824	0	
20–24 yrs	11,546	0		10,833	0	
25–29 yrs	11,345	0		11,296	0	
30–34 yrs	12,438	1	4.02 (95% CI: −7.12–15.16)	13,012	0	
35–39 yrs	16,139	0		16,384	0	
40–44 yrs	19,950	2	5.01 (95% CI: −4.81–14.84)	19,940	0	
45–49 yrs	18,380	3	8.16 (95% CI: −4.90–21.22)	18,030	0	
50–54 yrs	16,262	6	18.45 (95% CI: −2.43–39.32)	16,239	4	12.32 (95% CI: −4.75–29.38)
55–59 yrs	13,380	18	67.26 (95% CI: 23.33–111.20)	13,999	1	3.57 (95% CI: −6.33–13.47)
60–64 yrs	11,326	25	110.37 (95% CI: 49.22–171.52)	12,156	3	12.34 (95% CI: −7.41–32.09)
**<65 yrs**	**182,613**	**55**	**15.06 (95% CI: 9.43–20.69)**	**180,564**	**8**	**2.22 (95% CI: 0.04–4.39)**
65–69 yrs	9,174	32	174.41 (95% CI: 89.02–259.79)	10,193	3	14.72 (95% CI: −8.83–38.26)
70−74 yrs	7,757	57	367.41 (95% CI: 232.77–502.05)	9,171	4	21.81 (95% CI: −8.41–52.03)
75–79 yrs	5,058	53	523.92 (95% CI: 324.97–722.88)	6,428	3	23.34 (95% CI: −14.00–60.68)
80–84 yrs	3,654	37	506.29 (95% CI: 276.17–736.42)	5,651	6	53.09 (95% CI: −6.97–113.15)
85–89 yrs	2,515	26	516.90 (95% CI: 236.64–797.16)	4,396	5	56.87 (95% CI: −13.61–127.35)
Mes 90 yrs	1,013	5	246.79 (95% CI: −58.76–552.34)	2,696	1	18.55 (95% CI: −32.86–69.65)
**≥65 yrs**	**29,171**	**210**	**359.95 (95% CI: 291.22–428.67)**	**38,535**	**22**	**28.55 (95% CI: 11.68–45.41)**
Total	**211,784**	**265**	**62.56 (95% CI: 51.91–73.21)**	**219,099**	**30**	**6.85 (95% CI: 3.38–10.31)**

*N*: number of cases of bladder cancer in 2018–2019. CR: crude incidence rate per 100,000 person-years. Yrs: years.

## Data Availability

The datasets used and/or analyzed during the current study are available from the corresponding author on reasonable request.
